The article "DMA, a Bisbenzimidazole, Offers Radioprotection by Promoting NFκB Transactivation through NIK/IKK in Human Glioma Cells" was retracted in 2020. Reasons: duplicated images; unreliable results or conclusions; concerns about the data; concerns about the images.

# DMA, a Bisbenzimidazole, Offers Radioprotection by Promoting NFκB Transactivation through NIK/IKK in Human Glioma Cells

**DOI:** 10.1371/journal.pone.0039426

**Published:** 2012-06-22

**Authors:** Navrinder Kaur, Atul Ranjan, Vinod Tiwari, Ritu Aneja, Vibha Tandon

**Affiliations:** 1 Dr B. R. Ambedkar Center for Biomedical Research, University of Delhi, Delhi, India; 2 Department of Chemistry, University of Delhi, Delhi, India; 3 Department of Biology, Georgia State University, Atlanta, Georgia, United States of America; Institut Gustave Roussy, France

## Abstract

**Background:**

Ionizing radiation (IR) exposure often occurs for human beings through occupational, medical, environmental, accidental and/or other sources. Thus, the role of radioprotector is essential to overcome the complex series of overlapping responses to radiation induced DNA damage.

**Methods and Results:**

Treatment of human glioma U87 cells with DMA (5- {4-methylpiperazin-1-yl}-2-[2′-(3, 4-dimethoxyphenyl)-5′-benzimidazolyl] in the presence or absence of radiation uncovered differential regulation of an array of genes and proteins using microarray and 2D PAGE techniques. Pathway construction followed by relative quantitation of gene expression of the identified proteins and their interacting partners led to the identification of MAP3K14 (NFκB inducing kinase, NIK) as the candidate gene affected in response to DMA. Subsequently, over expression and knock down of NIK suggested that DMA affects NFκB inducing kinase mediated phosphorylation of IKKα and IKKβ both alone and in the presence of ionizing radiation (IR). The TNF-α induced NFκB dependent luciferase reporter assay demonstrated 1.65, 2.26 and 3.62 fold increase in NFκB activation at 10, 25 and 50 µM DMA concentrations respectively, compared to control cells. This activation was further increased by 5.8 fold in drug + radiation (50 µM +8.5 Gy) treated cells in comparison to control. We observed 51% radioprotection in control siRNA transfected cells that attenuated to 15% in siRNA NIK treated U87 cells, irradiated in presence of DMA at 24 h.

**Conclusions:**

Our studies show that NIK/IKK mediated NFκB activation is more intensified in cells over expressing NIK and treated with DMA, alone or in combination with ionizing radiation, indicating that DMA promotes NIK mediated NFκB signaling. This subsequently leads to the radioprotective effect exhibited by DMA.

## Introduction

Exposure to IR, as well as other stresses, triggers several complex signaling pathways, including DNA damage recognition and repair, induction of cell cycle checkpoints, senescence and/or apoptosis [1], [2]. Damage to other cellular components, such as the cell membrane, mitochondria, endoplasmic reticulum, and non-DNA constituents of chromatin, may also initiate or modify stress signaling in response to IR. Some of the important pathways responding to radiation include the ATM/P53pathway, MAPK cascades and NFκB activation, as well as signaling events initiated at the cell membrane and within the cytoplasm [3]. The signalling loop concept exists as activation of membrane and cytoplasmic kinases in response to DNA damage inflicted by ionizing radiation. A complex of nuclear factor-κB (NFκB), essential modulator and ataxia telangiectasia- mutated kinase activated by genotoxic agents is sent to cytoplasm, prompting nuclear translocation of the active transcription factor NFκB. In parallel, linear signalling pathways are initiated in the cytoplasm, mostly by reactive oxygen species (ROS), resulting in NFκB activation and nuclear translocation. The choice of NFκB activation pathway and the extent of activation of various pathways may be influenced by the relative degree of damage inflicted by genotoxic agents in the nuclear and cytoplasmic compartments. The ultimate pattern of cellular response is determined by availability, abundance and localization of the proteins participating in the signal transduction. The fate of damaged cells depends on the balance between pro- and antiapoptotic signals. In this decisive life or death choice, the transcription factor NFκB has emerged as a prosurvival actor in most cell types [4], [5]. Early microarray analysis of radiation exposed human cells revealed several novel radiation-induced genes, including FRA1 and ATF3, which encode important transcription factors and require functional p53 for radiation responsiveness [6]. Signaling through MAP kinase pathways can also contribute to the molecular response to radiation exposure. It has been shown that ERK 1/2 pathway has been involved in the upregulation of EGR-1 [7] and VEGF [8] expression in the presence of ionizing radiation mediated by activator protein 1(AP-1) which may lead to further neovascularization and proliferation of glioblastoma cells.

The complexity of signaling that occurs following exposure to IR allows flexibility in determining the ultimate fate of damaged cell or tissue. Competition between p53 and NFκB has been shown to sway the balance between apoptosis and survival of irradiated cell. The NFκB-inducing kinase (NIK) is a mitogen-activated protein kinase kinase kinase that potently induces NFκB. Although the upstream receptor remains uncertain, downstream NIK signaling leads to marked activation of the IκB kinases (IKKs) [9], which phosphorylate IκBα, leading to its rapid ubiquitination and degradation by the 26S proteasome. Inactive NFκB/IκB may continuously shuttle between the cytoplasm and nucleus; however, degradation of IκBα allows DNA binding by the liberated NFκB complex and promotes target gene expression [10]–[12]. NFκB plays a key role in cytokine and growth factor signaling, serving to regulate the expression of panoply of genes that mediate inflammatory, anti-apoptotic, and proliferation or differentiation signaling [13], [14].

Hoechst 33342 had been shown to protect genomic DNA against radiation-induced damage. It was reported that the radioprotective activity may be improved by the addition of electron-donating substituents to the ligand [15]–[17]. On the other hand, inhibition of topoisomerase as well as chromatin structure dependent DNA repair by Hoechst 33342 lead to a higher level of residual DNA damage, resulting in a higher level of cytogenetic damage, cell cycle perturbations, and genomic instability, thereby enhancing cytotoxicity [18]. Therefore, development of DNA binding ligands that afford a radioprotective effect without causing mutagenic and cytotoxic effects can play a significant role in biological radioprotection. Here we report the radioprotective effects of two minimally cytotoxic synthetic disubstitutedbenzimidazoles-DMA (Fig. 1A) and TBZ (5-{4-methylpiperazin-1-yl}-2-[2′{2′′-(4-hydroxy-3-methoxyphenyl)-5′′-benzimidazolyl}-5′-benzimidazolyl]. Their radiomodifying effects were investigated on BMG1, a human glioma cell line exposed to Co-60 gamma irradiation by determining cell survival and cell proliferation compared with that of the parent compound, Hoechst 33342. Results from radiation induced growth inhibition showed that DMA & TBZ afforded 84% and 100% radioprotection respectively in human brain glioma cells (BMG1 cells) [19]. Both ligands quench free radicals in isolated free radical system suggesting their dual mode of action against radiation induced damage to DNA. Our data indicate a 2-fold protection by DMA [20], which acts through altering DNA structure and free radical quencher both, as compared to Hoechst, which had shown free radical quenching only. The cell survival assay on four cell lines; human epithelial cancer cells (Hela), human breast cancer cell line (MCF7), human glioma cell line (U87), Human embryonic kidney cell line (HEK) was done previously in our laboratory [21].

**Figure 1:** Effect of DMA on survival of HDF, MCF10A and U87 cell lines. (A) Structure of the DNA minor groove binding ligand DMA –5-(4-methylpiperazin-1-yl)-2-[2′-(3,4-dimethoxyphenyl)-5′-benzimidazolyl] benzimidazole.(B) Effect of varying concentrations of DMA on metabolic viability studied by MTT assay in exponential growing HDF,MCF10A and U87 cells at 24 h, (C) At 48 h (D) At 72 h.Values are mean (±SD) of three independent experiments.Statistical significance by T-test p<0.05.

Herein, we sought to gain insights on the enhanced radioprotective efficacy and noncytotoxicity of DMA (Fig. 1A). Microarray hybridization and protein expression analysis by 2D PAGE revealed large number of genes that are regulated in response to DMA and/or ionizing radiation. Real time quantitation of the identified proteins and headers confirmed differential regulation. On the basis of our results we propose the involvement of NFκB inducing kinase as the regulator of gene expression modulation in response to DMA and/or ionizing radiation.

## Results

### DMA Exerts Reduced Cytotoxicity

In our earlier publications, we have already established that DMA is a radioprotector and it protects the human brain glioma cells (BMG1) from radiation and it is less cytotoxic to several cancer as well as transformed cell lines [19]. In view of above, it became imperative to evaluate the cytotoxicity of DMA in normal cells. We examined the cytotoxicity of DMA in primary human dermal fibroblasts (HDF) and near normal mammary epithelial cells (MCF10A) over a wide range of concentrations (0.1–150 µM) up to 72 h post DMA treatment. Interestingly, the IC_50_ of DMA in HDF and MCF10A could not be determined up to 72 h suggesting that DMA is less cytotoxic to normal cells in comparison to cancerous cells and can be developed as safe therapeutic agent. In addition to it we have measured the toxicity of DMA in U87 cell line also as it possess wild type p53 status and have been taken up as a system for studying irradiation and cytoprotective effects previously.The half maximal inhibitory concentration (IC_50_) of DMA was found to be 100 µM at 24 h in U87 cells (Fig. 1B, C, D).

### Differential Gene Expression in Response to DMA and Radiation Treatment in U87, Human Glioma Cells

PANTHER gene expression tool was used to classify the differentially expressed genes affected by the three different treatment conditions in U87 human glioma cells, when compared to non-treated control, into specific pathways (Table 1). A total of 30 pathways were found to be differentially expressed in U87 cells treated with DMA, radiation and DMA+radiation (P<0.005). In DMA treated U87 cells, higher percentage of genes modulated were from the General transcription by RNA polymerase I (45%), General transcription regulation (8.82%), Cell cycle (13.636%), Transcription regulation by bZIP transcription factor (9.43%), Insulin/IGF pathway-MAP kinase cascade (14.28%), Insulin/IGF pathway-protein kinase B signaling cascade (13.48%) pathways as compared to radiation alone. On the contrary, higher percentages of genes modulated in the radiation treated U87 cells were from oxidative stress response (11.66%), p53 pathway (10.619%), p53 pathway feedback loops 2 (11.538%) as compared to DMA or DMA+ radiation with respect to control (Untreated cells).

**Table 1:** List of pathways and number of genes in each pathway identified in U87 cells in three different treatment conditions DMA (50 µM), radiation (8.5 Gy) and DMA+ radiation (50 µM +8.5 Gy) after 4 h by Microarray hybridization studies.

Pathways	DMA	Radiation	DMA+Radiation
VEGF signaling pathway	14	6	10
Oxidative stress response	5.5	13	7.4
FAS signaling pathway	14.6	17.4	9
Glutamatereceptor group II pathway	14	8.8	8.8
PDGF signaling pathway	13.8	10.5	13.5
Cadherin signaling pathway	13	12	11
Nicotinic acetylcholine receptor signaling	14.2	10	15
IGF pathway-protein kinase B signaling	14.2	10	10
IGF pathway-MAP kinase cascade	15	12.3	9
Ras pathway	14.8	4	8
Ubiquitin proteosome pathway	15	15	15
p53 pathway feedback loops 2	10	12	6
bZIP transcription factor	10	4.6	4.6
Interleukin signaling pathway	11.2	7.2	8
TGF-beta signaling pathway	14.8	9	8
p53 pathway	5.4	10.8	7.5
PI3 kinase pathway	10.6	6	6.4
Salvage pyrimidine ribonucleotides	22	14.4	7.5
Cell cycle	14	5	12.2
Wntsignaling pathway	10.6	10.6	11
Apoptosis signaling pathway	5	11	8
Integrin signaling pathway	10.6	6	6
General transcription regulation	9	5	6.4
Notch signaling pathway	7	4.6	4.6
Cytokine signaling pathway	10.4	5.7	6
Synaptic vesicle trafficking	21.4	18	15.8
DNA replication	28	14.6	14.6
FGF signaling pathway	6.2	3	2
General transcription	45	15	35

From these pathways, a number of representative differentially expressed genes identified are given in Table 2. Two important NFκB signaling related genes - CREB3L4 and TRERF, were induced in DMA treated cells. Other related transcription factors- HIF1A, ASCC3 and CREBBP were found to be upregulated in response to DMA treatment. MAP3K14 (NFκB inducing kinase) was upregulated in DMA and DMA + radiation treated cells.

**Table 2:** List of genes differentially regulated in U87 cells 4 h after treatment with DMA (50 µM), radiation (8.5 Gy) and DMA + radiation (50 µM+8.5 Gy).

Accessionnumber	Genesymbol	Gene Name	Function	DMA	Radiation	DMA+Radiation
NM_130898	CREB3L4	cAMP responsive element binding protein3-like 4	regulation of transcription,DNA-dependent	**4.03**	1.55	1.65
AF297872	TRERF1	transcriptional regulating factor 1	Transcription regulation	**4.9**	0.54	6.45
NM_005902	ASCC3	Activating signal cointegrator 1 Complexsubunit 3	Transcription regulation	**5.290**	0.86	1.68
AC004760	CREBBP	CREB binding protein	mRNA transcriptionregulation	**2.18**	0.18	1.92
BC012527	HIF1A	hypoxia-inducible factor 1, alpha subunit	Transcription activation	0.981	0.909	**5.075**
AC008105	HIF!A	Mitogen activated protein kinasekinasekinase 14	Positive regulation ofNFkB cascade	**4.236**	0.456	**1.375**
NM_004045	ATOX1	ATX1 antioxidant protein 1 homolog (yeast)	response to oxidative stress	**0.137**	0.82	**0.11**
NM_012111	AHSA1	AHA1, activator of heat shock 90 kDa proteinATPase homolog 1(yeast)	response to stress	**0.146**	1.5	**0.17**
NM_005742	PDIA6	Protein disulfide isomerase family A, member 6	protein folding	**0.15**	0.84	**0.15**
BC015484	CALB2	calbindin 2, 29 kDa (calretinin)	calcium ion binding	**0.131**	1.07	**0.12**
NM_007236	CHP	calcium binding protein P22	calcium ion binding	0.52	1.05	**0.086**
NM_002155	HSPA6	heat shock 70 kDa protein 7 (HSP70B)	unfolded protein response	**0.441**	0.91	**0.493**
NM_006597	HSPA8	heat shock 70 kDa protein 8	unfolded protein response	**0.327**	0.74	**0.474**
BC024034	HSPA9	heat shock 70 kDa protein 9 (mortalin)	unfolded protein response	**0.395**	0.93	0.59
NM_005347	HSPA5	heat shock 70 kDa protein 5(glucose-regulated protein 78 kDa	unfolded protein response	**0.06**	0.77	**0.118**
NM_002157	HSPE1	heat shock 10 kDa protein 1 (chaperonin 10)	unfolded protein response	1.07	**3.74**	1.03
NM_145046	CALR3	calreticulin 3	unfolded protein binding	1.28	**5.09**	1.04
BT019740	PRDX1	peroxiredoxin 1	peroxiredoxin 1	0.97	1.22	**0.002**
BT020007	PRDX3	peroxiredoxin 3	redox regulation	0.66	0.70	**0.169**
NM_012473	TXN2	thioredoxin 2	response to hypoxia	1.49	1.32	**0.067**
NG_005218	HSP90AA3P	heat shock 90 kDa protein 1, alpha-like 1	Chaperone	1.43	1.74	**0.071**
NM_006993	NPM3	nucleophosmin/nucleoplasmin, 3	nucleic acid binding	**0.20**	1.27	**0.105**
BC009623	NPM1	nucleophosmin (nucleolarphosphoproteinB23, numatrin)	nucleic acid binding	**0.27**	1.55	**0.16**
NM_006472	TXNIP	thioredoxin interacting protein	response to oxidative stress	**0.18**	1.29	**0.202**
NM_001540	HSPB1	heat shock 27 kDa protein-like2 pseudogene; heat shock 27 kDa protein	unfolded protein response	**0.44**	1.66	**0.464**
NM_022121	PERP	PERP, TP53 apoptosis effector	induction of apoptosis	**0.28**	3.87	**0.244**
BC022307	ATM	similar to Serine-protein kinase ATM (Ataxia telangiectasia mutated)	DNA Repair	0.69	0.84	**0.194**
NM_001924	GADD45A	growth arrest and DNA-damage-inducible, alpha	DNA Repair	**0.329**	1.24	0.64
NM_015675	GADD45B	growth arrest and DNA-damage-inducible, beta	DNA Repair	**0.113**	0.64	**0.378**
NM_006705	GADD45G	growth arrest and DNA-damage-inducible,gamma	DNA Repair	**0.177**	0.94	**0.206**
NM_007233	TP53BP1	TP53 activated protein 1	Response to DNA damage	**0.119**	0.783	0.51
NM_005657	TP53AP1	TP53 binding protein 1	Response to DNA damage	**0.14**	2.41	1.13
NM_006034	TP53I11	TP53 inducible protein 11	Response to stress	**0.203**	1.06	0.69
NM_002578	PAK3	p21 (CDKN1A)-activated kinase 3	protein serine/threoninekinase activity	**0.154**	1.16	**0.17**
NM_020168	PAK6	p21 (CDKN1A)-activated kinase 6	protein serine/threoninekinase activity	**0.22**	1.22	**0.21**
NM_004964	HDAC1	histone deacetylase 1	regulation of transcription,DNA-dependent	**0.216**	0.69	**0.35**

(D = 50 µM DMA treated cells, R = 8.5 Gy irradiated cells, D+R = 50 µM DMA+8.5 Gy treated cells; Fold change values in red indicate upregulation in comparison with control untreated cells (2 fold and above); Fold change values in green indicate downregulation in comparison with untreated control (0.5 fold and.

### 2D PAGE Reveals Modulation of Protein Expression in Response to DMA and Radiation Treatment

A total of 19 proteins were identified and observed as differentially regulated (upregulated or downregulated) in response to DMA, radiation and DMA+ radiation with respect to control (untreated cells) by 2D PAGE and ESI-MS/MS analysis (Fig. 2 and Table S1, S2).

**Figure 2:** One representative image of 2D PAGE of the proteome of U87, cells in response to DMA, radiation and DMA+radiation treatment. Protein spots showing differential expression in the DMA, radiation and DMA+ radiation at 4 h time point, an average of three replicates (data derived from replicate wells) are annotated with arrows and numbers. The numbers given in this figure denote the 19 differentially expressed proteins identified by 2D PAGE and ESI-MS/MS analysis. The serial numbers 1–19 in table S1 denote the protein spots numbered in Figure 2. The left hand side spots are of protein marker.

These differentially expressed proteins belonged to four different categories- chaperones and folding catalysts (HSP70, CALR, TRX, PRX2, PDIA3); structural proteins (UBCEP80, H2B1, ACTG, TPM4, VIM, FABPE); Single stranded nucleic acid binding proteins (NPM1,PCBP1); Glycolytic pathway enzymes (PGM, ENO1,TPI, PARK7,NACA). Since most of these proteins are interacting partners, a pathway construction was attempted by online available sources (KEGG, NCBI). This pathway converged onto three mitogen activated protein kinases–MAP3K3, MAP3K7 & and MAP3K14 (Fig.3).

**Figure 3:** Pathway construction based on the proteins identified from 2D PAGE and ESI-MS/MS Analysis . Genes/proteins identified from proteomic data analyses were categorized into pathways based on NCBI, OMIM, KEGG and Gene Cards. Colour boxes represent the proteins identified by ESI-MS/MS- chaperones and folding catalysts (HSP70, CALR, TRX, PRX2, PDIA3); structural proteins (UBCEP80, H2B1, ACTG, TPM4, VIM, FABPE); Single stranded nucleic acid binding proteins NPM1,PCBP1); Glycolytic pathway enzymes (PGM, ENO1,TPI); PARK7,NACA. Blue boxes indicate interacting partners not identified by ES-MS/MS but are common between the identified proteins as interacting partners. Red arrows indicate that the proteins identified belonging to common categories and possessing common interacting partners converge onto MAPK signal transduction pathway.

### Relative Quantitation of Gene Expression of 2D PAGE Identified Proteins by Real Time PCR

Out of the total genes identified from 2D page, a total of 5 genes of MAP kinase pathway were quantitated by RT PCR. Out of the five MAP kinase pathway genes, YWHAZ and MAP3K14 (NIK) were found upregulated in response to DMA and DMA + radiation treated cells. However, no effect was observed in response to irradiation only. In the case of MAP3K3, MAP3K7 and MAP3K10, no significant differential expressions were observed in all the treatment conditions. Similarly, NFκB (RelA subunit) was observed to be differentially regulated in DMA and DMA+ radiation treated cells in comparison to radiation alone (Fig. 4).

**Figure 4:** Relative quantitation of gene expression for MAPK pathway genes in U87 cells. U87 cells were treated with 50 µM DMA and/or 8.5 Gy ionizing radiation. RNA samples were prepared 4 h after treatments. YWHAZ (14-3-3 zeta), MAP3K3 (Mitogen activated protein kinase kinasekinase 3), MAP3K7 (Mitogen activated protein kinase kinasekinase 7), MAP3K14 (Mitogen activated protein kinase kinase 14), MAPK10 (Mitogen activated protein kinase 10) and NFκB (Nuclear Factor Kappa B/Rel A subunit) were quantitated by Real Time PCRusing RNA samples from U87 glioma cell line. Values represent Mean±S.D.(*indicates statistical significance by T-test, *p<0.05).

### DMA Potentiates NFκB- Inducing Kinase Mediated Activation of IKKα and IKKβ

The phosphorylation of both IKKα and IKKβ were not observed in control and radiation treated U87 cells, transfected with control siRNA through western blot experiments (Fig.5). However, in response to DMA and DMA + radiation, phosphorylated IKKα was observed. Phosphorylated IKKβ was also observed albeit to a weaker extent (Fig. 6). Over expression of NFκB- inducing kinase by transfecting U87 cells with p3XFLAG CMV10 NIK plasmid potentiated the activation of IKKα and IKKβ in DMA treated cells (Fig. 7). Minimal level of IKKα phosphorylation was observed in control cells, with no phosphorylation of IKKβ being detected. In radiation treated cells, activation of both IKKα and IKKβ was not observed. In response to DMA and DMA+radiation, phosphorylated form of both IKKα and IKKβ was detected. In all the samples, detection of IκBα was abrogated concurrent with observation of phosphorylated form of either IKKα or IKKβ (Fig.7). Transfection of U87 cells with siRNA-NIK and subsequent knock down of NFκB- inducing kinase expression gave a different response (Fig.6). In all the treated samples, phosphorylated form of both IKKα and IKKβ was not observed. However, total IKKα, IKKβ and IκBα were detected at all the time points. There was no change observed in total protein levels of both IKKα and IKKβ, following DMA and TNF-α stimulation.

**Figure 5:** Effect of transfection with control-siRNA on the phosphorylation of IKKα and IKKβ. U87, human glioma cells were transiently transfected with control-siRNA. Cells were induced with 10 ng/ml TNF-α for 0,5,10,20,40,60 min and treated with DMA (50 µM) and/or irradiated at 8.5 Gy. Phosphorylation of IKKα, IKKβ was observed in DMA treated cells, alone or in combination with IR.

**Figure 6:** Effect of transfection with siRNA-NIK on the phosphorylation of IKKα and IKKβ. U87, human glioma cells were transiently transfected with siRNA-NIK. Phosphorylation of IKKα, IKKβ was absent concurrent with equivalent expression of IκBα in response to both DMA and radiation treatment.

**Figure 7:** Effect of NFκB inducing kinase overexpression on the phosphorylation of IKKα and IKKβ. U87, human glioma cells were transiently transfected with p3XFLAG CMV10 NIK. Phosphorylation of IKKα, IKKβ was advanced in NIK overexpressing cells as compared to siRNA transfected cells in response to DMA treatment, alone or in combination with IR.

### siRNA -NIK Knock down Abrogates DMA-induced Radioprotection in Transfected Cells

*In vitro* cell proliferation assay was used to study radioprotective ability of DMA in siRNA-NIK transfected and control siRNA transfected cells with or without radiation [22]. As shown in Fig. 8, the percentage of radioprotection by DMA in control siRNA transfected cells with respect to drug only control at 24, 48 and 72 h was 51%,30% and 16% respectively while in siRNA-NIK transfected cells the percentage of radioprotection by DMA was 15%, 18% and 10% at 24, 48 and 72 h respectively.

**Figure 8:** Radioprotection afforded DMA studied by proliferation kinetics assay in Control siRNA and siRNA-NIK transfectedU87 cells. (A) U87 cells (Control siRNA transfected) were treated with 50 µM DMA and 8.5 Gy Radiation. Post treatment cells were seeded in 6 well plates seeded at 8000 cells/cm2, and their proliferation kinetics was studied at 24 h intervals following trypsinization and counting total cells per well using a hemocytometer. (B) U87 Cells post siRNA-NIK oligonucleotide transfection were treated with 50 µM DMA and 8.5 Gy Radiation. Post treatment cells were seeded in 6 well plates seeded at 8000 cells/cm2, and their proliferation kinetics was studied at 24 h intervals following trypsinization and counting total cells per well using a hemocytometer. Values are mean (±SD) of three independent experiments.Statistical significance by T-test p<0.05.

### DMA does not Perturb Cell Cycle

To further study the effect of DMA on cell cycle, we examined the cell cycle in control siRNA transfected as well as siRNA-NIK transfected U87 cells. We have observed normal cell cycle in control siRNA treated cells, whereas cells did show a strong G2 check point after irradiation alone. There was clear G2 phase accumulation (18.9%) at 6 h after exposure to 8.5 Gy, which was increased till 18 h (34.5%), came near to normal at 24 h (22.3%) (Fig. 9E, G). There was no strong/significant G2 check point observed after DMA (50 µM) treatment in control siRNA treated cells, but in DMA + radiation treated cells we have observed a significant G2-M (43.5%) arrest than the irradiated cells (34.5%) at 18 h(Fig. 9E, G). The delay in cell cycle progression is probably exploited by the cells to perform DNA repair, and as a consequence to reduce the adverse effects of radiation, such as cell killing and induction of mutations. The cell cycle analysis of siRNA-NIK transfected cells also showed strong G2 check point after radiation treatment (11.9% at 0 h, 13.3% at 3 h, 18.6% at 6 h, 30.3% at 12 h, 43.6% at 18 h and 29.7% at 24 h), whereas the G2 check point response in DMA + radiation treated cells was almost similar to radiation only treated group reassuring that the activity of DMA is diminished in NIK abrogated cells (Fig 9. F, H).

**Figure 9:** DMA attenuates radiation induced apoptosis in U87 through NIK. (A) Apoptosis analysis of control siRNA transfected U87 cells at 3 h, 6 h in different treatment condition i.e. 50 µM DMA, radiation (8.5 Gy) and DMA (50 µM) + Radiation (8.5 Gy). Percentage of apoptosis is defined by % of cells that are Annexin V^+^ and Annexin V ^+^PI^+^. (B) Apoptosis analysis of siRNA-NIK transfected U87 cells at 3 h, 6 h in different treatment condition i.e. 50 µM DMA, radiation (8.5 Gy) and DMA (50 µM) + Radiation (8.5 Gy). Percentage of apoptosis is defined by % of cells that are Annexin V^+^ and Annexin V ^+^PI^+^. (C) Percentage of Annexin V^+^ and Annexin V ^+^PI^+^.positive cells in control siRNA transfected U87 cells at, 3 h,6 h, and 24 h in different treatment condition i.e. 50 µM DMA, radiation (8.5 Gy) and DMA (50 µM) + Radiation(8.5 Gy). (Data Not shown for 6 h and 12 h for only DMA and only radiation treatment condition). (D) Percentage of ofAnnexin V^+^ and Annexin V ^+^PI^+^.positive cellssiRNA-NIK transfected U87 cells at 3 h, 6 h, and 24 h in different treatment condition i.e. 50 µM DMA, radiation (8.5 Gy) and DMA (50 µM) + Radiation (8.5 Gy).(Data Not shown for 6 h and 12 h for only DMA and only radiation treatment condition). (E) Time course graphs showing the progression of cell cycle of control siRNA transfected U87 cells at 0, 3, 6, 12, 18 and 24 h in different treatment condition i.e. 50 µM DMA, radiation (8.5 Gy) and DMA (50 µM) + Radiation(8.5 Gy). (F) Time course graphs showing the progression of cell cycle of siRNA-NIK transfected U87 cells at 0, 3, 6, 12, 18 and 24 h in different treatment condition i.e. 50 µM DMA, radiation (8.5 Gy) and DMA (50 µM) + Radiation(8.5 Gy). (G) Cell cycle progression of control siRNA transfected U87 cells showing % G2-M fraction at 0, 3, 6, 12, 18 and 24 h in different treatment condition i.e. 50 µM DMA, radiation (8.5 Gy) and DMA (50 µM) + Radiation(8.5 Gy). (H) Cell cycle progression of siRNA-NIK transfected U87 cells showing % G2-M fraction at 0, 3, 6, 12, 18 and 24 h in different treatment condition i.e. 50 µM DMA, radiation (8.5 Gy) and DMA (50 µM) + Radiation(8.5 Gy).

The Annexin V assay showed lot of early and late apoptotic events in radiation treated U87 cells upto 24 h. The percentage apoptosis kept increasing in radiation treated cells till 24 h in a significant manner. In DMA + radiation treated cells the total (35% at 3 h, 30% at 6 h and 18% at 24 h) of early and late apoptotic cells were observed less in comparison to radiation treated cells only (45% at 3 h, 6 h and 24 h data not shown) (Fig 9. A, C). But in NIK knocked down cells the apoptotic events were almost similar in radiation (60% at 3 h, 6 h and 24 h data not shown) as well as DMA + radiation treated cells (58% at 3 h, 52% at 6 h, and 52% at 24 h), suggesting that NIK plays a role in the radioprotection activity of DMA. (Fig 9. B, D). Recently, there is a report where role of NIK was implicated in cell survival, supporting our observation [23].

### DMA Affects NFκB Activation in a dose Dependent Manner

TNF-α induced NFκB dependent reporter gene transcription assay showed no activation of NFκB in control and radiation treated cells. To confirm that the activation of NFκB was specifically caused by DMA, a series of concentration of DMA (0, 10, 25, 50 µM) was used in cells co-transfected with pNFκB-Luc (0.2 µg/well) and pRenilla (0.02 µg/well) and induced with 20 ng/ml TNF-α (Fig. 10). The results showed that NFκB activation was promoted in a dose-dependent manner by DMA. From 10 to 50 µM, a concentration dependent increase in induction of NFκB activation was observed in response to DMA. Higher induction of NFκB activation was observed in 50 µM DMA treated cells exhibiting a fold change of 3.62. However, NFκB activation was abrogated in U87 cells following irradiation. In DMA + radiation treated cells, activation of NFκB was again dose dependent with higher activation occurring in 50 µM + radiation treated cells i.e.; 5.77 fold as compared to control cells.

**Figure 10:** Luciferase assays for NFκB activation in U87 cells. Cells were co-transfected with pNFκB-Luc and pRenilla. After 24 h, cells were irradiated (8.5 Gy) with or without DMA treatment (50 µM) and stimulated with TNF-α (20 ng/ml) for 4 h prior to cell lysis. Luciferase activity was determined to quantify NFκB transcription activity. Relative Luciferase activity (RLA) for NFκB activation was increased in DMA treated cells compared with irradiated or control cells. The triplicate samples were used and the data was presented as mean±SD from three independent experiments. (*indicates statistical significance by T-test, *p<0.00001).

### Identification of NFκB Inducing Kinase as the Candidate Gene

From microarray hybridization and data analysis (Table 2), three important NFκB signaling related genes - CREB3L4, ASCC3 and TRERF were induced in DMA treated cells. It has been reported that CREB3L4 is a bZIP transcription factor that localizes to the membrane of endoplasmic reticulum and plays a role in cell homeostasis. It also has transcriptional activation activity from NFκB regulatory elements [24]. Another related transcription factor-ASCC3 was found to be upregulated in response to DMA treatment. ASCC3 has been reported to exist as a steady-state complex associated with three polypeptides, P200, P100, and P50, which stimulates transactivation by serum response factor (SRF), activating protein 1 (AP-1), and Nuclear factor kappaB (NF-kappaB) through direct binding to SRF, c-Jun, p50, and p65; and relieves the transrepression between nuclear receptors and either AP-1 or NF-kappaB. TRERF is another important transcription factor that has been observed to interact with CREBBP and EP300 resulting in a synergistic transcriptional activation of CYP11A1. Expression of HIF1A was found to be increased in DMA + radiation treated cells. It was reported that activation of HIF1A requires recruitment of transcriptional coactivators such as CREBBP and EP300.It also binds to core DNA sequence 5′-[AG] CGTG-3′ within the hypoxia response element (HRE) of target gene promoters. Since CREBBP is a coactivator of P300/CREB, increase in its expression would oppose the proapoptotic function of p53. Expression of HIF1A [25] was increased in DMA + radiation treated cells. Hence, we observed upregulation of NFκB inducers and effectors from microarray and real time PCR results. The key signaling molecule observed as upregulated was NFκB inducing kinase, which subsequently leads to mobilization of NFκB from cytosol to the nucleus thereby activating the nuclear targets and hence the transactivation of downstream genes. Thus, activation of NFκB inducing kinase in DMA treated cells perhaps may explain counteraction of radiation- induced damage.

## Discussion

On the basis of microarray hybridization and data analysis of differentially regulated genes following pathways were observed to be differentially regulated on DMA and ionizing radiation treatment in U87 cells – Apoptosis pathway, Chaperones and folding catalysts, Transcription regulator, oxidative stress response cell cycle, signal transduction and p53 pathway. Two prominent NFκB signaling related genes - CREB3L4 and TRERF were induced in DMA treated cells. We observed expression of a number of NFκB signaling related genes (MAP3K14, CREBBP, CREB3L4, TRERF, ASCC3 and HIF1A) to be regulated in response to DMA from Microarray hybridization and data analysis. Thus, the concerted action of CREB3L4, TRERF, ASCC3 and HIF1A induces CREB/p300 and NFκB results in opposition of proapoptotic response and increase in transcriptional activation.

Regulation of MAP3K14, CREB3L4, ASSC3, HIF1A points towards the activation of the NFκB mediated signaling pathway. Marked increase in NFκB activation in DMA treated cells indicates promotion of cell survival and proliferation. Simultaneously, downregulation of HSP70, stress responsive gene as observed in cells treated with DMA could further lead to reduction in inhibition of the NFκB inducing kinase, since HSP70 blocks NFκB activation via inhibition of both I kappa B kinase (IκK) activation and subsequent degradation of I kappa B alpha (IκBα) [26], [27]. Induction of NFκB inducing kinase subsequently leads to mobilization of NFκB from cytosol to the nucleus thereby activating the nuclear targets and hence the transactivation of downstream genes. This as an effect could result in the suppression of misfolded protein response, apoptosis and regulation of gene expression to ensure enhanced cell survival (Fig. 11).

**Figure 11:** Proposed hypothesis for the mechanism of action of DMA. From gene expression analysis, important inducers of NFκB-CREB3L4, TRERF, ASCC3, HIF1A and MAP3K14 were observed to be activated. Moreover, HSP70 was found to be downregulated which inhibits NFκB activation at the level of I kappa B Kinase. Suppression of chaperones, folding catalysts, stress responsive genes in DMA treated cells further adds onto cellular proliferation. Thus, in cells treated with DNA minor groove binding ligand DMA, induction of NFκB inducing kinase and related transcription factors converges onto the propagation of the pro-survival signal.

In addition following p53 pathway genes were downregulated in DMA treated cells- PERP,ATM,GADD45A,GADD45B,GADD45G,TP53BP1,TP53AP1,TP53I11,PAK3,PAK6,HDAC1. In cells treated with DMA alone, we observed simultaneous activation of NFκB and downregulation of p53 responsive genes (Table 2). p53 is generally a proapoptotic transcription factor, while NFκB promotes resistance to programmed cell death. The NFκB had an ability to suppress p53 transactivation and thus inhibitthe transcriptionally dependent induction of apoptosis by p53.Sequestration of p300 and CBP competitively; is likely to be understood as an increasingly common mechanism regulating inducible gene expression. It has been shown that p53 and RelA (NFκB) can bind p300 and CBP competitively, the answer may lie in the utilization of different p300/CBP complexes, being used by distinct subsets of DNA-binding proteins, thus functionally separating them and limiting cross talk to certain regulatory families of transcription factors [28], [29].Hence, the activity of NFκB may directly oppose the proapoptotic function of p53 activation through competition for the p300/CREB-binding protein transcriptional coactivator complexes. Thus, treatment with DMA leads to activation of NFκB inducers and effectors and provides comparatively enhanced radioprotective efficacy.

In cells treated with DMA alone, we observed simultaneous activation of NFκB and CCNB2, CASP8, THBS1 and CCNG2 of p53 pathway were downregulated. Similarly BAX, CDK4, CCNG1, SESN1were found to be upregulated in DMA+ radiation treated U87 cells with no change in radiation alone. In our earlier work, we had observed that DMA modulates radiation damage to DNA through free radical quenching, which was supported by observing regulation of a number of genes in apoptotic pathway in U87 cell line. TNFRSR1A, CASP8, PIK3R5, BCL1, CAPN1 were found to be downregulated in DMA treated cells. Since these genes are the central components of apoptotic response their downregulation in response to DMA further implicates the absence of DNA damage. Thus, treatment with DMA leads to activation of NFκB inducers and effectors and provides comparatively enhanced radioprotective efficacy.

In summary, suppression of expression of stress activated genes, absence of activation of DNA damage responsive genes, and over expression of signal transduction genes as well as transcription regulation factors may be possible reasons behind the radioprotective ability of this molecule as observed by attenuated DNA damage at the cellular level.

A total of 19 proteins were identified as differentially expressed and categorized into four pathways using KEGG-chaperones and folding catalysts, structural proteins, single stranded nucleic acids binding proteins and metabolic enzymes on the basis of 2D PAGE analysis of U87 cells. Protein expression of five chaperones and folding catalysts was observed to be altered- HSP70, CALR, TRX, PRDX, and PDIA. A number of structural proteins were also identified as differentially expressed- UBCEP80, H2B1, ACTG, TPM4, VIM and FABPE. Two single stranded nucleic acids binding proteins-NPM and PCBP1 were found to be upregulated in radiation treated cells, however, in cells treated with DMA only, were found to be normally expressed. Enzymes belonging to the glycolytic pathway found to be differentially regulated were- PGAMB, ENO1 and TPI. Pathway construction using online available resources, on the basis of identified proteins and their interacting partners led onto the identification of the headers (MAP3K14, MAP3K7 and MAP3K3) that could be involved in modulation of radiation response by DMA in U87 cells (Fig. 3). RT PCR was performed to verify changes in expression of 21 genes. 19 genes were chosen from 2D PAGE results and two more i.e.; MAP3K14, header of the pathway constructed by us on the basis of 2D PAGE results, and NFκB a downstream gene of MAP3K14 were also included for real time study. Relative quantitation of above genes(data not shown for all genes) suggested modulation of a number of genes - HSP70, TXN, PDI, CALR, PRDX, YWHAZ, NPM1, PCBP1, MAP3K14, NFκB, H2B1.

RT PCR experiments validated modulation of YWHAZ, MAP3K14, NFκB in MAP kinase pathway genes in all treatment conditions (Fig. 4). YWHAZ belongs to the family of 14-3-3 proteins that are pivotal regulators of intracellular c-Abl localization and of the apoptotic response to genotoxic stress [30]. Upregulation of this gene in response to DMA, both alone and in combination with IR shows regulation of cell cycle machinery by DMA. NFκB is known as a proinflammatory transcription factor and is now confirmed as an antiapoptotic and prosurvival force in the most cell types [31]–[33]. This gene was upregulated in DMA and DMA + radiation treated cells, thus implicating the activation of pro-survival genes in response to DMA. MAP3K14, an upstream kinase was upregulated in DMA and DMA+ radiation treated cells. It has been reported that MAP3K14 binds to Traf2 and stimulates NFκB activity [34]–[36].

Amifostine, along with other thiol-containing drugs, such as N-acetylcysteine (NAC), mesna, and oltipraz, which have been approved for clinical use as radioprotector, are capable of participating in intracellular reductive/oxidative processes that have broad clinical implications. These include effects on the activation of redox-sensitive transcription factors, alteration of gene expression, and modification of protein activities. Amifostine, NAC and oltipraz activate the redox-sensitive transcription factor NFκB in the absence of oxidative stress–inducing agents [37]–[41]. DNA-binding motifs for NFκB were found in the promoter regions of more than 150 genes, many of them involved in inflammatory processes and the survival response [14]. NFκB is an inducible transcription factor that plays an essential role in the expression of a number of gene families that include cytokines and their receptors, cell adhesion molecules, growth factors, and antioxidant genes [42]. A number of reports have described the activation of NFκB by reducing agents, when present at mM concentrations, such as NAC, dithiothreitol, 2-mercaptoethanol 2-ME, oltipraz, and amifostine [38]–[40], [43]. It has been reported that exposure of glioma cells to mM concentrations of WR-1065 significantly protected these cells from the cytotoxic and mutagenic effects of ionizing radiation [44], [45]. The Putrescine, spermidine, and spermine have each been reported to participate in the activation of NFκB and to enhance its binding to nuclear response elements (NREs) [46]. The underlying mechanism of action is not attributed to changes in oxidative stress, but rather to the ability of these positively charged molecules to activate NFκB and affect structural/conformational changes in DNA that facilitate an enhanced binding of NFκB to its NRE sequences.

On the basis of above results, we identified NFκB inducing kinase as the candidate gene affected by DMA. Western blots results suggested that DMA affects NIK mediated NFκB activation. In cells overexpressing NIK, DMA promoted activation and phosphorylation of IKKα and IKKβ, although extent of phosphorylation of IKKβ was weaker than IKKα. Activation of IKKα and IKKβ in DMA treated samples, alone or in combination with radiation, was concurrent with degradation of IκBα. As compared to cells treated with control-siRNA, activation was advanced in time in cells over expressing NIK. On the contrary, cells in which the NIK expression was knocked down by siRNA-NIK, no activation and phosphorylation of IKKα and IKKβ was observed in response to DMA, alone or in combination with IR. Luciferase reporter assay confirmed dose dependent induction of NFκB activation.

Biochemically the apoptotic process is first recognized by alterations of surface lipid composition, in that, phosphotidylserine, which is normally on the inner leaflet of plasma membrane, translocates to the outer leaflet, which can be easily measured by fluorescent labeled Annexin V binding assay. An impermeable dye propidium iodide, cannot enter the cells unless the cells are under late apoptosis, when membrane permeability is compromised. This can be quantified in large population of cells by flow cytometry. The control siRNA (untreated) cell culture contained very few apoptotic cells (6.5%) (Data not shown), which were assigned as the background cell death due to stress during normal cell culture. We found that in DMA (50 uM ) treated U87 transfected with control siRNA, resulted in 9% early apoptotic cells within 24 h, but radition (8.5 Gy ) treated cells showed 45% early apoptotic cells within 3 h which were reduced to 35% at 3 h, 30% at 6 h and 18% at 24 h in DMA + radiation treated cells. The U87 cells transfected with siRNA-NIK, showed 60% apoptotic cells after irradiation (8.5 Gy) at 3 h time point, which were consistant to 58% at 3 h, 52% at 6 h and 52% at 24 h in DMA + radiation treated siRNA-NIK transfected cells. The Annexin V assay showed that DMA causes a very few apoptotic events in U87 cells, hence DMA can be proposed as a safe molecule. This result is in concurrence of our earlier results in which DMA was observed less cytotoxic in comparison to parent molecule Hoechst 33342, a free radical quencher, no significant DNA damage was observed through comet assay [20].

We observed higher RQ value of NFκB in DMA treated cells as compared to DMA+radiation treated cells in RT-PCR. However, in luciferase reporter assay higher activation of NFκB was observed in DMA+radiation treated cells as compared to DMA treated cells in luciferase reporter assay. From a RT-PCR experiment only the transcript level is measured, but luciferase reporter assay takes into account promoter binding dependent activation and/or post transcriptional modification or transactivation. Hence, reporter assay is a more direct study of the NFκB protein level in response to DMA and/or radiation treated cells. Therefore, ultimately we observed higher activation of NFκB in DMA + radiation treated cells.

We observed absence of IKKα and IKKβ activation and phosphorylation as well as subsequent NFκB activation in irradiated cells. Reactive oxygen species (ROS) increase first promotes NFκB activation by triggering NIK activation, which usually leads to prosurvivaltranscriptional events. However, as ROS become overwhelming, the nuclear environment is shifted from reductive to oxidative, which inhibits activation of NFκB and other transcriptional factors by preventing them from binding to DNA. As a consequence, the prosurvival transcription activity is abolished [47]. This increased ROS then leads to shift in survival/death control.

We examined the effect of NIK inhibition by siRNA on the proliferation of U87 cells in DMA treated cells in the presence and absence of radiation. We observed a significant decrease of 36% in Radiation protection in siRNA- NIK treated cells as compared to control siRNA treated U87 cells at 24 h. The complete absence of radioprotection was not observed as we had already established that DMA, has a dual mode of action against radiation [20], it also acts as free radical quencher. The parent analogues Hoechst 33258 & 33342 were well identified as free radical quencher, generated directly or indirectly by IR [18], [48].

These results are in the agreement with our microarray, real time and western blot results suggesting that the radioprotective effect of DMA is NIK mediated. Collectively, our data suggests that, one of the primary targets of DMA is NIK. We may conclude that radioprotective effect of DMA is due to NIK mediated NFκB activation leading irradiated cells to antiapoptotic and prosurvival pathway, one of the plausible mechanisms of action of DMA as a radioprotector.

Amifostine is converted into active form in normal cells by alkaline phosphatase which is inactive in an acidic environment of tumors making it a selective drug for normal cells. The major side effects of amifostine are transient hypotension, flushing, somnolence, metallic taste and transient hypocalcaemia. Also amifostine effect will be reduced in tumor cells due to hypoxia state [49]. On the contrary, our molecule DMA has dual mode of action i.e.;free radicals quenching and binding to DNA which makes it a better molecule [19]. Our cytotoxicity data suggest that DMA is more toxic to cancerous cells then normal cells. Abnormal vasculature of cancerous cells can be one of the possible modes of differential uptake of DMA in cells. Thus our correlation of NIK and DMA in U87 cells can be further elucidated for clinical importance in normal cell lines. NIK/IKK mediated NFκB activation is at a pivotal role for promoting pro-survival in cells hence the clinical relevance of this study; as further work in normal cells and animal model experiments can lead to development of a novel radioprotector with enhanced survival and radioprotection with less cytotoxicity which is a major drawback among most other well known radioprotectors. It was suggested that coactivation of prosurvival ATM/ERK/NFκB pathway offer an effective therapeutic approach for enhancing radiation tolerance in human skin cells [50] . Several groups have tested the effects of NFκB inhibitors on cellular radiosenstivity and shown that the NFκB activity is necessary for enhancing cell survival under high dose radiation. In addition, it was also observed that IKKβdependent NFκB activation provides radioprotection to the intestinal epithelial cells [51]. Similarly our results suggests that, DMA activates the NIK/IKKα/IKKβ mediated NFκB activation providing protection to cells from higher γ –radiation doses.

## Materials and Methods

### Cell Culture

The human glioma cell line U87 was obtained from the National Centre for Cell Science (Pune, India). MCFA10A was obtained from American Type Culture Collection (ATCC) USA and HDF cells were obtained from Dermatology department at Emory University School of Medicine, Atlanta, GA, USA. These cells lines were maintained according to the ATCC recommendations at 37°C, 5% CO_2_, in DMEM supplemented with 10% heat inactivated FCS, 50 units/ml penicillin, 50 µg/ml streptomycin. Cells were cultured, grown until ∼ 80% confluent, trypsinized and seeded in 90 mm culture dishes for 24 h before experiments.

We have used U87 cells for the present study due to number of reasons. Earlier, we have showed in BMG1 cell line (Glioma cells) that DMA is a noncytotoxic radioprotector. We measured the radio sensitivity of U87cells with a standard clonogenic assay [52] and found U87 cells were medium sensitive to radiation and survival of these cells, after radiation is higher than other cells. U87 cell lines possess wild type p53 status and have been taken up as a system for studying irradiation and cytoprotective effects previously [53]–[56]. Amifostine, a radioprotector which is in clinical trial and lot of previous work was done and validated with U87 cells.

### DMA and Exposure Conditions

DMA was synthesized in our laboratory as described previously [19]. IC_50_ for DMA was determined at 100 µM in U87 cells. Radioprotection survival assay was performed using increasing dose of DMA from 0–100 µM concentration at four different radiation doses- 2, 5, 8.5 and 10 Gy respectively (data not shown). The radiation dose (8.5 Gy) and drug dose (50 µM) was determined by clonogenecity assay at increasing ligand concentration as well as increasing radiation dose. From the clonogenecity assay it was observed that, 50 µM at 8.5 Gy provided best radioprotection. At higher radiation dose most of the cells died in DMA untreated cells (control cells). Hence, in this study all the experiments were performed at 50 µM DMA with or without 8.5 Gyradiation. Stock of DMA was prepared in methanol and further dilution to 1 mM was done using DMEM. This solution was then filtered & sterilized and U87 cells were subjected to DMA treatment at a final concentration of 50 µM for 1 h. Four treatment conditions were studied- control (untreated), ligand treated (50 µM DMA), radiation treated (8.5 Gy radiation) and ligand + radiation treated (50 µM DMA+8.5 Gy radiation).

### Irradiation Procedure

1 h subsequent to DMA treatment, cells were exposed to 8.5 Gy γ- irradiation (1.3 Gy/min dose rate) using Co-60 source (Institute of Nuclear Medicine and Allied Sciences, Delhi, India). Following irradiation, cells were incubated for 4 h in a 5% CO_2_ humidified incubator. Trypsin was used to detach the cells. Cells were centrifuged, washed twice in 1X PBS (pH 7.4) and processed for further sample preparation.

### Metabolic Viability Assay

Exponentially growing U87, HDF and MCF10A cells were plated at cell densities 3000 cells per well in 96-well tissue culture plates. After 24, 48 and 72 h cells were treated with increasing concentrations of DMA i.e.; 0.1–150 µM. Cytotoxicity was measured by MTT assay according to the manufacturer’s instructions (Promega, Madison, WI, USA). The experiments were performed in triplicate and repeated thrice. The percentage survival was calculated as percent of 570 nm OD of DMA treated cells to that of DMA untreated control cells with 630 nm OD as reference.

Percentage survival  =  (Calculated difference between measurement and reference OD of DMA treated cell/Calculated difference between measurement and reference OD of DMA untreated cell) X 100.

### Microarray Hybridization and Analysis

Total RNA was extracted from the cell lines using Tri Reagent (Ambion), digested by DNase (RNase free, MBI Fermentas) and purified using Qiagen™ RNeasyminikit. RNA concentration and purity was determined using NanoDrop spectrophotometer (Thermo Fischer, MA, USA). RNA quality was evaluated by Agilent 2100 BioAnalyzer (Agilent Technologies Inc., Palo Alto, CA), and RNA integrity number (RIN) was found9.0. The 5.0 µg of total RNA was used for amplification using the Express Art® mRNA amplification kit. Amplified aRNA (aminoallyl antisense RNA) was then labelled with Cy3™ post-labelling reactive dye pack (GE Healthcare, United Kingdom) at RT. 20 µg of the labelled aRNA in 200 µl of Ocimum’sHyb buffer was denatured at 95°C for 3 min and 100 µl was used for hybridization performed at 50°C for 2 h on Tecan HS 4800 automated Hyb station. Human 40 KA and 40 KB OciChip™ (OcimumBiosolutions, Hyderabad) consisting of 20160 and 19968 spots respectively were printed on Corning® epoxy coated glass slides using Omnigrid (Gene Machines). Oligos were printed using spotting buffer A at 50% humidity and 22°C. The RNA samples were then hybridized and processed according to OciChip™ 40K Array manual specifications. For each treatment condition, three independent experiments were performed. Hybridized Chips were scanned using Affymetrix 428™ array scanner at three different PMT gains setting- 40, 50, 60. Data were collected and stored as Tiff images and further analyzed using Imagene software. The mean background intensity was subtracted from the mean target intensity to produce the signal intensities. Initial dataset that consisted of 40,320 probes was filtered to exclude quality control (QC) probes and empty spots. The data was transformed using log-transformation and median absolute deviation was performed. After normalization, genes in the treatment groups with at least two-fold change in expression were considered as up-regulated or downregulated in comparison to non treatedcells (control). To determine significant proportions of differentially expressed genes within functional groups, the hypergeometric probability P was calculated. P<0.005 was considered significant. The gene expression values generated were analyzed using online available tool- PANTHER (www.pantherdb.org).All microarray data are MIAME compliant and the raw data has been deposited in Gene Expression Omnibus (GEO) with accession number GSE30043. The individual accession number of genes is mentioned in the table 2.The links for access to microarray data submitted to the GEO are as mentioned below:

http://www.ncbi.nlm.nih.gov/geo/query/acc.cgi?acc=GSE30043(U87 cell line).

### Protein Extraction, 2D PAGE and Image Analysis

Protein samples were prepared from cells harvested from DMA and radiation treated cells as described elsewhere [57]. Cells were lysed in lysis buffer containing 8 M urea, 0.5% (w/v) CHAPS, 50 mMTris, 0.2% (w/v) Bio-Lyte 4/7, 50 mM DTT, 1 mM PMSF, 1 mM EDTA, 10% (v/v) Glycerol and 1–2 µg/µl protease inhibitor cocktail (Bio-Rad, Hercules, CA), vortexed at RT for 10 min, incubated on ice for 15 min and centrifuged in a microcentrifuge at 12,000 rpm for 10 min. The protein concentration was determined using the Bradford method with bovine serum albumin as a standard. The supernatant was combined with 200 µl of rehydration Buffer (Bio-Rad) containing 8 M urea, 2% CHAPS, 50 mM DTT, and 0.2% (w/v) Bio-Lyte 4/7 ampholytes, before isoelectric focusing. First dimensional separation of proteins (200 µg of protein in 200 µl) was performed on Ready Strip IPG strips (pH 4/7, 11 cm; Bio-Rad) for a total of 30,000 V-hours. The second dimensional separation was performed on a 12% acrylamide gel following DTT reduction and IAA alkylation. The gels were subsequently stained with Coomassie Brilliant Blue R250 and scanned using a Gel Documentation System (Alpha Imager) at 300 dpi and saved as a gray scale tiff file. Images were analyzed using Bio-Rad’s PD Quest software. The protein pattern differences between the control, radiation treated and DMA treated samples were elucidated by analyzing images from each sample using Bio-Rad’s PD Quest software. For each treatment sample, three independent experiments were performed. The software assigns a standard spot parameter number based on the quality and type of spots. Using the Gaussian Model during Test, quality and quantity values were assigned to spots based on total quantity in valid spots following normalization.

### In-Gel Trypsin Digestion and ESI-MS/MS

Differentially regulated protein spots were excised from gels and destained using 50 mM Ammonium Bicarbonate and 50% Acetonitrile. Spots were subsequently dried using 100% Acetonitrile, speed dried under vacuum and digested with 20 ng/µl trypsin (Promega Trypsin Gold, Mass Grade) in 25 mM Ammonium Bicarbonate overnight at 37°C. Peptides were extracted from gel pieces using 60% Acetonitrile, 0.5% Formic Acid. Samples were purified using a C_18_ microbed column (Millipore ZipTip). Samples were then analyzed by ElectroSprayIonization tandem mass spectrometry (ESI-MS/MS; Applied Biosystems Q-Star XL) at a voltage of 1200 V. Sample spectra were acquired using TOF MS and tandem mass spectral data as well as using an IDA (information dependent acquisition) feature in the Analyst QS software. The IDA experiments selected multiply charged precursors (charged state from 2 to 5) for fragmentation with an intensity threshold of 10 counts per second. Precursor ions were excluded for 60 seconds using a window of 6 atomic mass units and collision energy settings were automatically determined by IDA based on *m/z* values.

### Database Queries and Protein Identifications

The acquired tandem mass spectral data were queried against protein database using the MASCOT search engine (version 1.8, Matrix Science Ltd., U.K.) with a mass tolerance of 100 ppm and one trypsin miscleavage. Carbamidomethylation of cysteine was set as variable amino acid modifications. For a given sequence, the EST analyzer searched NCBInr protein database to identify a homologous protein (the best hit of BLASTX search), then used the homologous protein to annotate the query sequence. Proteins with MOWSE scores equal to the accepted significant threshold (determined at 95% confidence level as calculated by MASCOT) were reported in this study.

### Pathway Construction

Online resources (NCBI, Gene Cards, OMIM and KEGG) were used to construct a pathway for proteins identified from 2D PAGE and their interacting partners. This pathway was utilized to identify the candidate genes.

### Real Time RT- PCR

The transcript levels of genes identified from 2D PAGE were analyzed for their expression by Real-Time Polymerase Chain Reaction (RT-PCR) using gene specific primers obtained from Sigma Aldrich (Table 3). RNA was isolated using TriReagent (Ambion), digested with DNase I (MBI Fermentas) and purified using Qiagen™ RNeasy mini kit. RNA samples were quantified using NanoDrop Spectrophotometer. The RIN was found to be 8.0.1 µg of RNA sample was converted into cDNA, and transcript levels were quantitated using Sybr Green I (Power Sybr Green I, Applied Biosystems) and Roche’s light cycler 480 instrument (LC_480_) according to manufacturer’s guidelines. β Actin gene was used as a internal control. Each experiment for samples was performed three times independently. The calculations and data analysis were done using the efficiency calibrated mathematical model for the relative expression ratio in real time PCR [58].

**Table 3:** Sequences of primers used for quantitation of gene expression.

S. No.	Gene	Primer sequences (FP- forward primer; RP-reverse primer)	T_m_ (°C)
1.	MAP3K3	FP-GAACTCCCCCTCACTGTTGARP-GAAGCAGGCACCTCTCTGTC	60.060.1
2.	MAP3K7	FP-CAAACAACTCCAAAGGCTCCRP-CTCCTCCTCCTCCTCGTCTT	59.759.9
3.	MAP3K14	FP-CCCTTCTCTCACAGCTCCATRP-ATGGAGGACAAGCAGACTGG	59.460.2
4.	MAPK10	FP-TTCACATCCAATGTTGGTTCARP-CAGGCCCATCTCAGATCTTC	59.859.7
5.	YWHAZ	FP-GAAGCATTGGGGATCAAGAARP-ACAAAAGACGGAAGGTGCTG	60.060.2
6.	NFκB	FP-CCACCTTTACGAGGACCTATTCCRP- CAGCACTCGCTCTCCATGAA	60.160.3

### Expression Vectors

The construct for NIK was obtained by cloning the requisite sequence into p3XFLAG CMV10 generously provided by Dr. P. C. Rath, School of Life Sciences, Jawaharlal Nehru University, Delhi. The construct of the NFκB-driven luciferase reporter gene and corresponding control construct for Renilla luciferase were kindly provided by Dr. Balram Ghosh, Institute of Genomics and Integrative Biology, Delhi.

### Transfection with Expression Vectors

The day before transfection, 6 well plates were seeded with 2×10^5^ cells/well in serum containing antibiotic free medium. The cells were incubated at 37°C in a 5% CO_2_ incubator overnight. For each well, plasmid was prepared in required volume of serum free medium. Transfectin™ Lipid Reagent (Bio-Rad, Hercules, CA) was prepared in serum-free medium. The DNA and Transfectin solutions were mixed together and incubated for 20 min at room temperature. DNA-Transfectin complexes were added directly to cells in serum-containing medium and swirled gently. Cells were incubated at 37°C in a 5% CO_2_ incubator. Additional media was added 4–6 h after addition of complexes. After 48 h, cells were harvested and assayed for protein expression.

### Cloning and Expression of NFκB Inducing Kinase

RNA was extracted from HEK cell line and cDNA was synthesized. The cDNA template of NFκB inducing kinase was amplified by PCR with sense primer NIK FP (5′-TCTAGAATGGCAGTGATGGAAATG-3′) and antisense primer NIK RP (5′-GGATCCTTAGGGCCTGTTCTCC-3′) using Phusion DNA polymerase (Finnzymes, Finland) and cloned into p3XFLAG CMV10. Subsequently, p3XFLAG CMV10 NIK plasmid was purified using EndoFree Plasmid Maxi Kit (QIAGEN™) according to manufacturer’s guidelines and dissolved in TE buffer (pH 7 to 8), before using for transfection. The transient transfection of the constructed plasmid was done by Transfectin Lipid Reagent (Bio-rad) according to the manufacturer’s guidelines.

### Knockdown of NIK using siRNA

In a 6 well tissue culture plate, human glioma (U87) cells were plated (2×10^5^ cells/well) in antibiotic free media supplemented with FBS. After 24 h, cells were transfected with siRNA-NIK (sc-36065, Santa Cruz Biotechnology Inc.) and control-siRNA (sc-37007, Santa Cruz Biotechnology Inc.) according to the manufacturer’s instructions. Knockdown of NIK was observed at 50 pM concentration of siRNA-NIK (Figure S1).

### Immunoblot Analysis

Human glioma (U87) cells were transfected with p3XFLAG CMV10- NIK, siRNA-NIK and control-siRNA using Transfectin (Lipid Reagent) according to manufacturer’s guidelines. For the experiment following transfections, cells were treated with 50 µM DMA for 1 h. Subsequently, cells were induced with TNF-α (10 ng/ml) for 0,5,10,20,40,60 min and irradiated at 8.5 Gy.Trypsin was used to detach the cells and the cells were collected, centrifuged at 2000 rpm for 2 min and resuspended in RIPA buffer (50mM Tris-HCl, pH 7.6, 150 mM NaCl, 1% sodium deoxycholate, 10% sodium orthovanadate and cocktail of protease inhibitors) on ice for 30 min. Following centrifugation at 25,000 g for 30 min, the supernatant was collected as total cell lysate and protein concentration was determined using Bradford’s Assay. Samples were prepared in SDS gel loading buffer (625 mM Tris pH 6.8, 10% SDS, 25% glycerol, 100 mM DTT and 0.015% bromophenol blue). Western blotting was performed using standard protocols with antibodies against human IKKα, IKKβ, IκBα, phospho-IKKα/IKKβ (180/181) (Santa Cruz Biotechnology Inc.) and horseradish peroxidase-conjugated mouse anti-human immunoglobulin (secondary antibody, Abcam). Detection was done by an enhanced chemiluminescence (ECL) system (Pierce).

### Proliferation Kinetics

U87 Cells post siRNA oligonucleotide transfections were treated with 50 µM DMA and 8.5 Gyradiation. Post treatment cells were seeded in 6 well plates at 8000 cells per well, and their proliferation kinetics was studied at 24 h intervals following trypsinization and counting total cells per well using a hemocytometer. Same experiment was done with control siRNA-transfected U87 cells. Percentage (%) radioprotection of cells was calculated by following formula.

% growth of Radiation treated cells  =  (Number of cells in Radiation treated cells/Number of cells in only DMA treated cells) X 100.

% growth of DMA+Radiation treated cells  =  (Number of cells in DMA+ Radiation treated cells/Number of cells in only DMA treated cells) X 100.

% Radioprotection  =  % growth of DMA+Radiation treated cells - % growth of Radiation treated cells.

### Cell-cycle Analysis

U87 cells (2×10^5^ cells/plate) in 60 mm plates, transfected with control siRNA and siRNA-NIK, were cultured and DMA, Radiation and DMA + Radiation treatment were given as described earlier. After irradiation, cells were collected after the incubation period of 0,3,6,12,18 and 24 h. After incubation cells were collected, washed twice with ice-cold PBS, and fixed in 70% ethanol. Cell pellets were stored at 4^o^C for 24 h. Cells pellets were washed twice with ice-cold PBS and stained with 0.5 mL of RNase (2 mg/mL) and 0.5 mL of propidium iodide (0.1% in 0.6% Triton X-100 in PBS) for 30 minutes in dark. Samples were then analysed on a FACSCalibur flow-cytometer (Becton Dickinson).

### Annexin-V Staining

U87 cells (2×10^5^ cells/plate) in 60 mm plates, transfected with control siRNA and siRNA-NIK, were cultured and DMA, Radiation and DMA +Radiation treatment were given as described earlier. After irradiation, cells were incubated for 3, 6, 12, 18 and 24 h (data not shown for 12 and 18h). Cells were collected by mild trypsinization and were pooled together with detached cells of respective group. Samples were prepared according to the manufacturer’s instructions (BD Pharmingen™ Annexin V: FITC Apoptosis Detection Kit I, Catalog Number 556547, USA) and the samples were subjected to flow cytometry analysis (Becton Dickinson).

### Luciferase Reporter Assay for NFκB Activity

The effect of DMA on TNF-α induced NFκB dependent reporter gene transcription was measured. Briefly, human glioma (U87) cells (2×10^4^ cells/well) were plated in 96 well plates. Next day cells were following serum starvation, cells were co-transfected with pNFκB-Luc (0.2 µg/well )and pRenilla (0.02 µg/well) using Transfectin™ Lipid Reagent (Bio-Rad, Hercules, CA) and β-galactosidase reporter vector (used as an internal control) according to the manufacturer’s instructions. pNFκB-Luc contains the firefly luciferase (*luc*) gene from *Photinuspyralis*. This vector also contains multiple copies of the NFκB consensus sequence fused to a TATA-like promoter (*P*_TAL_) region from the Herpes Simplex Virus thymidine kinase (HSV-TK) promoter. After endogenous NFκB proteins bind to the kappa (κ) enhancer element (GGGAATTTCCGGGAATTTCCGGGAATTTCCGGGAATTTCCGGGAATTTCCGGGAATTTCC), transcription is induced and the reporter gene is activated. Twenty four hours after transfection, U87 cells were treated with DMA (0,10,25,50 µM) for 1 h prior to irradiation at 8.5 Gy. Following irradiation, induction with TNF-α (20 ng/ml) was done for 4 h to induce NFκB driven luciferase expression. Subsequently, cells were assayed for reporter activity using Dual™ Luciferase Reporter Assay System (Promega) according to the manufacturer’s guidelines.The relative luciferase activity was calculated by normalizing results with the β –galactosidase expression.

### Statistical Analysis

Data are expressed as means ±SD. Statistical significance among groups was determined using the Student t test and the differences were considered significant at P<0.05.

## Supporting Information

Figure S1 **Knock down of NFκB inducing kinase gene expression using siRNA against NFκB inducing kinase.** (A) Lanes 1-5 - RT-PCR with siRNA treated cells with NFkB inducing kinase primers (control, 20 pM siRNA-NIK,50 pM siRNA-NIK,80 pM siRNA-NIK, NTC); Lanes 6-10- RT-PCR with siRNA treated cells with ACTB primers (control, 20 pM siRNA-NIK,50 pM siRNA-NIK,80 pM siRNA-NIK, NTC); M (DNA ladder). (B) Lanes 1-5 - RT-PCR with control siRNA treated cells with NFkB inducing kinase primers (control, 20 pM siRNA-NIK,50 pM siRNA-NIK,80 pM siRNA-NIK, NTC) Lanes 6-10- RT-PCR with siRNA treated cells with ACTB primers (control, 20 pM siRNA-NIK,50 pM siRNA-NIK,80 pM siRNA-NIK, NTC); M (DNA ladder).
(TIF)

Table S1 **Differentially regulated proteins identified by 2D PAGE and ESI-MS/MS analysis.**
(DOCX)

Table S2 **MS/MS analysis of reported proteins.**
(DOCX)
